# FTX Regulated miR-153-3p/FOXR2 to Promote Cisplatin Resistance in Ovarian Cancer

**DOI:** 10.1155/2022/2318170

**Published:** 2022-05-23

**Authors:** Ming Liu, Jingwei Peng

**Affiliations:** Department of Gynecologic Oncology, Shandong Cancer Hospital and Institute, Shandong First Medical University and Shandong Academy of Medical Sciences, Jinan 250117, China

## Abstract

**Purpose:**

The present study was aimed at exploring the role of FTX in cisplatin (DDP) resistance in ovarian cancer (OC).

**Methods:**

QPCR was applied to evaluate mRNA expression in OC tissue and cells. CCK-8 assay was conducted to evaluate cell proliferation. Transwell chamber assay was performed to evaluate invasion of SKOV3/DDP cells. The protein expression was evaluated via western blot assay. Flow cytometry was performed to evaluate the apoptosis of SKOV3/DDP cells.

**Results:**

The expression of FTX in DDP-resistant cells was observably higher in contrast to DDP-sensitive cells and normal ovarian cells. FTX was higher expressed in DDP-resistant tissues by comparison with DDP-sensitive tissues. Knockdown of FTX obviously suppressed the proliferation ability invasion ability of SKOV3/DDP cells. Knockdown of FTX obviously enhanced apoptosis of SKOV3/DDP cells. miR-153-3p was proved to be directly regulated by FTX via the luciferase reporter assays. By comparison with normal cells, miR-153-3p was lower expressed in OC cells. miR-153-3p was lower expressed in SKOV3/DDP cells in contrast to SKOV3 cells. More interestingly, FTX reversed the inhibiting influence of miR-153-3p on cisplatin resistance of OC cells. Moreover, miR-153-3p was proved to directly regulate FOXR2. Knockdown of miR-153-3p attenuated the inhibitory influence of knockdown FOXR2 on cisplatin resistance of OC cells.

**Conclusion:**

FTX regulated miR-153-3p/FOXR2 to promote cisplatin resistance via inhibiting the apoptosis and promoting the viability and invasion in OC.

## 1. Introduction

In China, the incidence rate of ovarian cancer (OC) is the third in all gynecological malignancies, accounting for 23% of the female reproductive tumors [1]. Patients with early ovarian cancer usually have some nonspecific symptoms, including pelvic pain, abdominal pain, and abdominal enlargement. These symptoms cannot clearly distinguish gynecological diseases from cancer [2]. Therefore, before the tumor metastasizes to the whole abdomen, there is no specific index to indicate that the patient has ovarian cancer. The prognosis of female patients with OC is directly related to the disease stage at the time of diagnosis [3]. In addition, chemotherapy resistance is also one of the direct causes of death. Therefore, the high mortality of OC is largely related to advanced diagnosis and chemoresistance [4]. Although the underlying mechanism leading to chemotherapy resistance is unclear, several factors are related to chemotherapy failure, including tumor heterogeneity, genetic instability, epigenetic changes, and tumor microenvironment.

Long chain noncoding RNAs (lncRNAs) are a kind of RNA, the length of which is greater than 200 bp, and have no protein coding function [5]. lncRNAs are essential in the occurrence and development of tumor by regulating different molecules such as mRNA and protein [6]. Despite the continuous progress in the research on the mechanism of tumor chemoresistance, we still know little about the mechanism mediated by lncRNA. lncRNA FTX is an essential factor in regulating the expression of Xist (X chromosome inactivation center) [7]. lncRNA FTX is closely relevant to the progression of malignant tumors [7–9]. However, the relationship between lncRNA FTX and chemoresistance of ovarian cancer has not been studied.

miRNAs widely exist in eukaryotes and are a kind of noncoding RNA with a length of 19-22 nucleotides, which regulate one or more genes [10]. miRNAs can affect the expression of a large number of proteins, including those cancer-related signaling pathways, such as apoptosis, migration, and metastasis [11]. miRNA regulates various normal physiological processes and is relevant to the occurrence and development of malignant tumors, including OC [12]. Therefore, more and more studies have been focusing on regulating the expression of miRNAs to regulate OC. Overexpression of miR-153-3p inhibited cell proliferation, migration, and induced apoptosis [13]. In addition, miR-153-3p increased the sensitivity of cancer cells to cisplatin [14]. Subsequently, studies focused on whether lncRNA affects tumor drug resistance by regulating mir-153-3p. lncRNA ROR enhanced the chemoresistance of osteosarcoma cells by regulating mir-153-3p [15].

This study was aimed at studying the influence of lncRNA FTX on the proliferation and invasion of cisplatin-resistant OC cells and then exploring the connection between lncRNA FTX and cisplatin resistance of ovarian cancer at the molecular level.

## 2. Materials and Method

### 2.1. Patient Specimens

After the patients received cisplatin (DDP) treatment, 23 DDP-resistant OC tissues, 23 DDP-sensitive OC tissues, and 23 normal tissues were acquired from patients in Shandong Cancer Hospital and Institute from February 2017 to January 2019. All patients received DDP treatment for 6 cycles. This study was approved by the ethics committee of Shandong Cancer Hospital and Institute. All patients participating in the trial have signed informed consent.

### 2.2. Cell Culture

SKOV3 and A2780 were contained in McCoy's 5A Media (Delf, China) with 10% FBS, while HOSE was contained in DMEM (Thermo Fisher, USA) containing 2% fetal bovine serum. All cells were contained at 37°C and 5% CO_2_. The drug-resistant cell lines were created by continuously culturing for 12 weeks with 8 *μ*M DDP.

### 2.3. Cell Transfection

The overexpression vectors of FTX, sh-FTX, sh-FOXR2 and their control, miR-153-3p mimics, anti-miR-153-3p, and their control were acquired from Genchem Biotechnology Co., Ltd. They were cotransfected into cells by Lipofectamine 2000 reagent (Thermo Fisher Scientific, USA).

### 2.4. Quantitative Real-Time PCR Analysis

The total RNA was extracted by TRIzol reagent (Invitrogen, USA) and was reverse transcribed to cDNA using the Takara reverse transcription kit (Takara, Japan). The mRNA expression was detected by SYBR Premix EX Taq II kit (Takara, Japan), and relative gene expression was analyzed by 2^-△△Ct^ method.

### 2.5. CCK-8 Assay

The cells were seeded at 5 × 10^3^ cells per well in 96-well plates. Five time gradients were set and the absorbance at 570 nm was measured at 0, 24, 48, and 72 h per well in the incubator.

### 2.6. Western Blot

Total protein was obtained using RIPA reagent (Corning, USA). Quantification was performed using a BCA kit. 10% SDS-PAGE was applied to separate protein. The protein bands were transferred to polyvinylidene difluoride (PVDF) membrane by semidry transmembrane method. Then, they were blocked using 5% skim milk for 2 h at 25°C. They were incubated overnight with appropriate amounts of the primary antibody (Corning, USA) at 4°C. PVDF membranes were washed the next day using Tris-HCL with Tween composite buffer and then were incubated for 2 h with the secondary antibody (Corning, USA). The gray-scale values scanned with Gel Imager were measured to quantify the expression of each protein.

### 2.7. Transwell Assay

200 *μ*L diluted Matrigel matrix (BD Biosciences, USA) was spread in a transwell chamber, which was placed in a 37°C, 5% CO_2_ incubator. 200 *μ*L cell suspension was added to the upper chamber, and 500 *μ*L DMEM medium (Gibco, USA) containing 10% FBS was added to the lower chamber. After 24 h, the cells crossing membrane were carefully erased with cotton swabs and were fixed with 4% paraformaldehyde and stained. The cell number was observed under an inverted microscope.

### 2.8. Luciferase Reporter Assay

The FTX wild-type luciferase reporter vector (FTX-WT) was constructed by Shanghai Biotechnology, and the binding site was also mutated to construct the FTX mutant luciferase reporter vector (FTX-MUT). The miR-153-3p mimics (or miR-NC) and FTX-WT (or FTX-MUT) were cotransfected to SKOV3/DDP cells using the Lipofectamine™ 2000 (Thermo Fisher Scientific, USA). Fluorescence intensity of firefly and sea kidney was examined via Dual-Luciferase Reporter Assay System.

### 2.9. Statistical Analysis

Analysis was conducted by SPSS19.0 statistical software. Comparisons between groups were performed by one-way ANOVA, and *P* < 0.05 was set as statistically significant.

## 3. Results

### 3.1. The Expression of LINC-FTX Decreased in DDP-Resistant OC Tissues and Cells

By comparison with normal tissues, FTX was higher expressed in OC tissues (Figure 1(a)). FTX was higher expressed in DDP-sensitive group by comparison with DDP-resistant group (Figure 1(a)). By comparison with normal cells, FTX was higher expressed in OC cells (Figures 1(b) and 1(c)). FTX was higher expressed in SKOV3/DDP and A2780/DDP cells by comparison with SKOV3 and A2780 cells (Figures 1(b) and 1(c)). The IC50 value of cisplatin obviously raised in SKOV3/DDP cells by comparison with SKOV3 cells (Figure 1(d)). CCK-8 assay suggested that viability of SKOV3/DDP cells was obviously higher by comparison with SKOV3 cells (Figure 1(e)).

### 3.2. FTX Promoted Cisplatin Resistance via Suppressing the Apoptosis and Enhancing the Viability and Invasion in OC Cells

Knockdown of FTX obviously decreased the FTX expression (Figure 2(a)). Knockdown of FTX obviously suppressed the proliferation ability (Figure 2(b)) and invasion ability (Figure 2(d)) of SKOV3/DDP cells. Knockdown of FTX obviously enhanced apoptosis of SKOV3/DDP cells (Figure 2(c)).

### 3.3. FTX Directly Regulated the Expression of miR-153-3p

miR-153-3p was predicted to might be regulated by FTX (Figure 3(a)). To prove miR-153-3p was regulated by FTX, the luciferase reporter assays were conducted. miR-153-3p decreased the luciferase activities of FTX-WT, while it showed unconverted effects on the FTX-MUT (Figure 3(b)). By comparison with normal cells, miR-153-3p expression was lower in OC cells (Figure 3(c)). miR-153-3p was lower expressed in SKOV3/DDP cells by comparison with SKOV3 cells (Figure 3(c)). Consistently, miR-153-3p expression increased in sh-FTX group (Figure 3(d)).

### 3.4. FTX Reversed the Inhibiting Influence of miR-153-3p on Cisplatin Resistance of OC Cells

miR-153-3p mimic observably increased miR-153-3p expression (Figure 4(a)). miR-153-3p obviously suppressed the proliferation ability (Figure 4(b)) and invasion ability (Figure 4(d)) of SKOV3/DDP cells and FTX reversed this impact. miR-153-3p obviously enhanced cell apoptosis and FTX reversed this impact (Figure 4(c)).

### 3.5. miR-153-3p Directly Downregulated FOXR2 Expression

FOXR2 was predicted to might be regulated by miR-153-3p (Figure 5(a)). In order to prove that FOXR2 was directly regulated by miR-153-3p, the luciferase reporter assays were performed. miR-153-3p decreased the luciferase activities of FOXR2-WT, while it showed unconverted effects on the FOXR2-MUT (Figure 5(b)). By comparison with normal cells, FOXR2 was higher expressed in OC cells (Figure 5(c)). FOXR2 was higher expressed in SKOV3/DDP cells by comparison with SKOV3 cells (Figure 5(c)). The expression of FOXR2 decreased in miR-153-3p mimic group (Figure 5(d)).

### 3.6. Silencing of miR-153-3p Attenuated the Inhibitory Effect of FOXR2 Knockdown on the Resistance of OC Cells to Cisplatin

The expression of FOXR2 obviously decreased following transfection with sh-FOXR2 (Figure 6(a)). FOXR2 knockdown obviously suppressed the proliferation ability (Figure 6(b)) and invasion ability (Figure 6(d)) of SKOV3/DDP cells and anti-miR-153-3p reversed this impact. FOXR2 knockdown obviously enhanced apoptosis of SKOV3/DDP cells and anti-miR-153-3p reversed this impact (Figure 6(c)).

## 4. Discussion

Many studies have recently indicated that lncRNA FTX is upregulated in multiple malignancies and affects the malignant behavior of tumor cells [7–9, 16]. lncRNA FTX could enhance cell proliferation and invasion in pancreatic cancer via binding to miR-513b-5p [17]. lncRNA FTX could enhance gastric cancer via regulating the downstream molecule miR-215 [18]. However, there are no reports on the relationship between lncRNA FTX and OC resistance. However, there is no report on the relationship between lncRNA FTX and OC chemoresistance. According to Liu's previous paper, FTX was higher expressed in adriamycin-resistant cells (U937/ADR and THP-1/ADR) by comparison with adriamycin-sensitive cells (U937 and THP-1) in acute myeloid leukemia (AML) [19]. We constructed OC DDP-resistant cell line SKOV3/DDP induced by cisplatin and found similar results. FTX expression in DDP-resistant cells was observably higher in contrast to DDP-sensitive cell and normal cells. FTX was higher expressed in DDP-resistant tissues by comparison with DDP-sensitive tissues. In addition, knockdown of FTX obviously suppressed the proliferation ability and invasion ability of SKOV3/DDP cells while enhanced apoptosis of SKOV3/DDP cells.

Next, we studied the mechanism of FTX promoting cisplatin resistance in OC cell. miR-153-3p was predicted to might be regulated by FTX, which was confirmed via the luciferase reporter assays. By comparison with normal cells, miR-153-3p was lower expressed in OC cells and SKOV3/DDP cells. The expression of miR-153-3p increased in sh-FTX group. More interestingly, FTX reversed the inhibiting effect of miR-153-3p. These results demonstrated that FTX promoted cisplatin resistance via regulating miR-153-3p. miR-153-3p was regulated by lncRNA and improves the sensitivity of multiple cancer to cisplatin [15, 20]. For instance, lncRNA ROR enhanced cisplatin resistance to osteosarcoma via binding to miR-153-3p [15].

Moreover, FOXR2 was proved to be directly regulated by miR-153-3p. FOXR2 increased the chemoresistance of bladder cancer [21]. The results of this study were consistent and found that the expression of FOXR2 is upregulated in SKOV3/DDP cells by comparison with SKOV3 cells. Inhibition of miR-153-3p attenuated the inhibitory effect of sh-FOXR2 on the resistance of OC cells to cisplatin. FOXR2 knockdown obviously suppressed the proliferation ability and invasion ability of SKOV3/DDP cells and anti-miR-153-3p reversed this impact. FOXR2 knockdown obviously enhanced apoptosis of SKOV3/DDP cells and anti-miR-153-3p reversed this impact.

In conclusion, FTX was higher expressed in DDP-resistant OC cells. FTX promoted cisplatin resistance via inhibiting the apoptosis and promoting the viability and invasion in OC cells. lncRNA FTX contributed to cisplatin resistance in OC by regulating FOXR2 via sponging miR-153-3p.

## Figures and Tables

**Figure 1:** The expression of FTX decreased in DDP-resistant OC tissue and cells. (a) FTX expression in tissues was detected via qPCR. *N* = 23. (b and c) FTX expression in OC cells was detected by qPCR. (d) IC_50_ value was evaluated via CCK-8 assay. (e) The cell viability was examined via CCK-8 assay. ^∗^*P* < 0.05.

**Figure 2:** Knockdown of FTX promoted cisplatin sensitive in SKOV3/DDP cells. (a) FTX expression was measured by qPCR. (b) The cell proliferation was examined via CCK-8 assay. (c) Cell apoptosis was measured via flow cytometry assay. (d) Cell invasion was examined via transwell assay. ^∗^*P* < 0.05.

**Figure 3:** FTX directly regulated miR-153-3p. (a) Predicted binding sites. (b) Inhibiting effect of miR-153-3p on luciferase activity of FTX-WT. (c and d) The expression of miR-153-3p was measured by qPCR. ^∗^*P* < 0.05.

**Figure 4:** FTX reversed the inhibiting influence of miR-153-3p on cisplatin resistance of OC cells. (a) The expression of miR-153-3p was measured by qPCR. (b) The cell proliferation was examined via CCK-8 assay. (c) Cell apoptosis was measured via flow cytometry assay. (d) Cell invasion was examined via transwell assay. I = miR-NC, II = miR-153-3p, III = miR-153-3p+Vector, IV = miR-153-3p+LINC-FTX. ^∗^*P* < 0.05.

**Figure 5:** miR-153-3p directly regulated FOXR2. (a) Predicted binding sites. (b) Inhibiting effect of miR-153-3p on luciferase activity of FOXR2-WT. (c and d) The protein expression of FOXR2 was measured by western blot in different cells line (c) and miR-153-3p group (d). ^∗^*P* < 0.05.

**Figure 6:** Silencing of miR-153-3p attenuated the inhibitory effect of FOXR2 knockdown on the resistance of OC cells to cisplatin. (a) The expression of FOXR2 was measured by western blot. (b) The cell proliferation was examined via CCK-8 assay. (c) Cell apoptosis was measured via flow cytometry assay. (d) Cell invasion was examined via transwell assay. I = sh-NC, II = sh-FOXR2, III = sh-FOXR2+anti-NC, IV = sh-FOXR2+anti-miR-153-3p. ^∗^*P* < 0.05.

## Data Availability

Data to support the findings of this study is available on reasonable request from the corresponding author.
